# Activated K-ras and INK4a/Arf Deficiency Cooperate During the Development of Pancreatic Cancer by Activation of Notch and NF-κB Signaling Pathways

This article has been retracted.

**DOI:** 10.1371/journal.pone.0020537

**Published:** 2011-06-03

**Authors:** Zhiwei Wang, Sanjeev Banerjee, Aamir Ahmad, Yiwei Li, Asfar S. Azmi, Jason R. Gunn, Dejuan Kong, Bin Bao, Shadan Ali, Jiankun Gao, Ramzi M. Mohammad, Lucio Miele, Murray Korc, Fazlul H. Sarkar

**Affiliations:** 1 Department of Pathology, Karmanos Cancer Institute, School of Medicine, Wayne State University, Detroit, Michigan, United States of America; 2 Division of Hematology and Oncology, Department of Internal Medicine, School of Medicine, Wayne State University, Detroit, Michigan, United States of America; 3 Sichuan College of Tranditional Chinese Medicine, Mianyang, Sichuan, People's Republic of China; 4 University of Mississippi Cancer Institute, Jackson, Mississippi, United States of America; 5 Department of Medicine and Department of Pharmacology and Toxicology, Dartmouth Medical School, Hanover, New Hampshire, United States of America; 6 Norris Cotton Comprehsive Cancer Center, Dartmouth-Hitchcock Medical Center, Lebanon, New Hampshire, United States of America; University of Nebraska Medical Center, United States of America

## Abstract

**Background:**

Pancreatic ductal adenocarcinoma (PDAC) is the fourth leading cause of cancer-related death in the United States, suggesting that novel strategies for the prevention and treatment of PDAC are urgently needed. K-ras mutations are observed in >90% of pancreatic cancer, suggesting its role in the initiation and early developmental stages of PDAC. In order to gain mechanistic insight as to the role of mutated K-ras, several mouse models have been developed by targeting a conditionally mutated K-ras^G12D^ for recapitulating PDAC. A significant co-operativity has been shown in tumor development and metastasis in a compound mouse model with activated K-ras and Ink4a/Arf deficiency. However, the molecular mechanism(s) by which K-ras and Ink4a/Arf deficiency contribute to PDAC has not been fully elucidated.

**Methodology/Principal Findings:**

To assess the molecular mechanism(s) that are involved in the development of PDAC in the compound transgenic mice with activated K-ras and Ink4a/Arf deficiency, we used multiple methods, such as Real-time RT-PCR, western blotting assay, immunohistochemistry, MTT assay, invasion, EMSA and ELISA. We found that the deletion of Ink4a/Arf in K-ras^G12D^ expressing mice leads to PDAC, which is in part mediated through the activation of Notch and NF-κB signaling pathways. Moreover, we found down-regulation of miR-200 family, which could also play important roles in tumor development and progression of PDAC in the compound transgenic mice.

**Conclusions/Significance:**

Our results suggest that the activation of Notch and NF-κB together with the loss of miR-200 family is mechanistically linked with the development and progression of PDAC in the compound K-ras^G12D^ and Ink4a/Arf deficient transgenic mice.

## Introduction

Pancreatic ductal adenocarcinoma (PDAC) is a highly aggressive malignant disease, which is ranked as the fourth leading cause of cancer-related death with a median survival of 6 months, and with an estimated 43,140 newly diagnosed cases and an approximately 36,800 deaths in the United States in 2010 [1]. It has been accepted that the development of PDAC occurs through the progression of precursor lesions such as pancreatic intraepithelial neoplasia (PanIN), ranging from low-grade PanINs (PanIN-1A, PanIN-1B) to high-grade PanINs (PanIN-2, PanIN-3) [2], [3]. PDAC has been shown to have multi-step molecular progression including high frequency of activating K-ras mutations and subsequent inactivation of p16^INK4a^, p53, SMAD4, p14ARF tumor suppressors and other additional genetic abnormalities in mouse models [4]–[6] and in human [7]. The most common K-ras mutation in human PDAC is on codon 12 (Kras^G12D^), which is related to the activation of GTPase activity. Therefore, several mouse models of PDAC have been generated by targeting a conditionally mutated K-ras^G12D^ to recapitulate the progression of PDAC [8]–[12]. One compound mouse model containing activated K-ras and Ink4a/Arf deficiency showed to cooperate in producing metastatic PDAC [13], [14]. However, the molecular mechanism(s) by which activated K-ras and Ink4a/Arf deficiency contribute to PDAC aggressiveness has not been fully elucidated.

In recent years, many signaling pathways including Notch pathway have been investigated and found to play important roles in PDAC [15]. Notch signaling has critical functions on the control of cell growth, differentiation, apoptosis, migration, invasion, and metastasis in PDAC [16]. Notch genes encode proteins which can be activated by interacting with a family of its ligands. To date, four Notch receptors (Notch1–4) and five ligands (Dll-1, Dll-3, Dll-4, Jagged-1, Jagged-2) have been identified [17]. Interestingly, it has been reported that the function of Notch signaling in tumorigenesis can be either oncogenic or oncosuppressive, and the function is also context dependent in PDAC [18], [19]. Notch signaling is frequently deregulated with up-regulated expression of Notch receptors and their ligands in PDAC [20]. We have shown that down-regulation of Notch-1 using specific siRNA was correlated with decreased proliferative rates, increased apoptosis, reduced migration, and decreased invasive properties of pancreatic cancer cells [21], [22]. Recently, it has been found that active Notch signaling can synergize with K-ras in PanIN initiation and progression to invasive adenocarcinoma [8], [23]. Inhibition of Notch signaling pathway resulted in the inhibition of tumor progression in a mouse model (K-ras, p53 L/+ mice) of PDAC [24]. More recently, Mazur et al. found that deficiency of Notch-2 stops PanIN progression, prolong survival through inhibition of Myc signaling in K-ras-driven pancreatic carcinogenesis [25]. Surprisingly, Notch-1 was recently found as a tumor suppressor in a model of K-ras-induced PDAC [18], suggesting that additional studies are required to determine the role of Notch signaling in PDAC.

Notch pathway has been reported to cross-talk with NF-κB, one of the major transcription factor associated with cell growth and apoptotic regulatory pathways in pancreatic cancer. Studies from our group revealed that Notch signaling could induce NF-κB activity in pancreatic cancer [21]. Recently, it was shown that NF-κB pathway is required for the development of tumors in a mouse model (K-ras, p53 L/L mice) of lung adenocarcinoma [26]. Moreover, it was found that genetic deletion of the NF-κB subunit p65 in a K-ras-induced lung cancer mouse model reduced lung tumorigenesis in the presence and in the absence of the tumor suppressor p53 [27]. However, it is largely uncertain whether NF-κB is necessary for K-ras-induced PDAC progression.

In the present study, we assessed the molecular alterations in mouse tumors developed in the compound transgenic mice with activated K-ras and Ink4a/Arf deficiency. Here, we show, for the first time, that deletion of Ink4a/Arf in K-ras expressing mice leads to PDAC, which is in part mediated through the activation of Notch and NF-κB signaling pathways. Moreover, we found alterations in the expression of miR-200 family, which could also play important roles in tumor development and progression of PDAC in the compound transgenic mice with activated K-ras and Ink4a/Arf deficiency.

## Results

### Notch signaling pathway is highly expressed in Pdx1-Cre;LSL-K-ras^G12D^;Ink4a/Arf mouse

To delineate the mechanistic role of mutated K-ras in the development and progression of PDAC, we assessed the expression of Notch pathway in the murine model. In this model, oncogenic K-ras (Kras^G12D^) is knocked-in into its own locus and transcriptionally silenced due to the insertion of a LoxP-Stop-LoxP element (LSL). When LSL- Kras^G12D^ mice are bred with transgenic mice which express Cre recombinase under the control of the Pdx1 promoter, expression of Cre recombinase in pancreatic progenitor cells allows the removal of the floxed transcriptional STOP cassette, leading to the activation of the oncogenic K-ras allele. In this model, there was no tumors readily found up to 30 weeks of age in LSL- K-ras^G12D^; Pdx1-Cre (we called KC in this manuscript) mice, consistent with previous study [13]. We also found no evidence of PDAC in the Ink4a/Arf; Pdx1-Cre (we called IC in this manuscript) animals up to an age of 24 weeks, similar to the observation documented by other groups [13]. However, all 25 mice from LSL- K-ras^G12D^; Pdx1-Cre; Ink4a/Arf (we called KCI for this manuscript) group were found to have pancreatic tumors ranging in diameter from 4 to 10 mm between 45 to 80 days (Fig. 1A). The compound KCI mice with tumors became moribund (Fig. 1A, survival curve). The tumors were confirmed by histopathologic examination (Fig. 1B). The Ki-67, a known proliferation marker, was highly expressed in KCI pancreatic tumors (Fig. 1B). It has been reported that Notch signaling pathway has critical roles in the development and progression of pancreatic cancer. Therefore, we assessed the expression of Notch genes in these transgenic mice tissues. It is important to note that we focused our studies on the cleaved Notch because it is the active functional form of Notch. Therefore, Notch in our all figure legends means active cleaved Notch. We found that Notch signaling was activated in the tumors of KCI mice when compared with the pancreata of KC and IC mice, respectively (Fig. 1C, D). The expression of Notch-2 and Notch-4 was up-regulated both at the mRNA and protein levels in KCI mice. However, Notch-1 expression showed no change and Notch-3 expression was increased only at the mRNA level in the tumors of KCI mice, suggesting that roles of Notch-2, and Notch-4 could be more important in progression of pancreatic cancer. We also found that all five Notch ligands were up-regulated in the tumors derived from the KCI mice (Fig. 2A, B). To confirm these results, we evaluated the expression of Notch downstream genes such as Hes-1 and Hey-1. We found that the expression of Hes-1 and Hey-1 was increased in the tumors of KCI mice (Fig. 2A, B), which was expected based on up-regulated expression of Notch-2, Notch-4 and their ligands.

**Figure 1:** Notch receptors are highly expressed in KCI mice. **A, Top** left panel: Tumor incidence in KCI mice (N>25). Control mice: KC and IC mice. Top right panel: Average length of tumors in KCI mice (N>20). **Bottom** panel: Kaplan-Meier pancreatic tumor-free survival curve for KCI mice and control animals. Control mice: combinations of KC and IC mice. **B, Top** panel: Microscopic examination of tumors derived from the KCI mice composed of cells which are forming ducts at places (red arrows). Focally tumor cells are in sheets. Cells are large, highly atypical, with large, pleomorphic nuclei and prominent 2–3 nucleoli (yellow arrows) per cell. Cytoplasm is eosinophilic with pale eosinophilic inclusions (green arrows) in few cells giving a rhabdoid feature to the cells. Surrounding stroma shows spindled cells with elongated nuclei (black arrows) and scattered inflammatory infiltrate comprising of neutrophils, lymphocytes and few plasma cells. **Bottom** panel: Ki-67 was highly expressed in tumors obtained from the KCI mice as assessed by immunohistochemistry. **C,** Notch signaling pathway was up-regulated at mRNA level as assessed by Real-time RT-PCR in tumors derived from the KCI mice. **D,** Notch pathway was highly expressed in tumors derived from the KCI mice as assessed by western blotting analysis and immunohistochemistry, respectively.

**Figure 2:** The expression of Notch ligands and NF-κB is upregulated in KCI mice. **A,** The expression of Notch ligands and Notch downstream genes was increased at mRNA level as assessed by Real-time RT-PCR in tumors derived from the KCI mice. **B,** The expression of Notch ligands and Notch downstream genes was highly expressed in tumors derived from the KCI mice as assessed by western blotting analysis. **C,** NF-κB p65 activity was increased in tumors derived from the KCI mice by ELISA. **D,** Left panel, NF-κB p65 DNA-binding activity is increased in tumors derived from the KCI mice as assessed by EMSA. Right panel, phospho-p65 was highly expressed in tumors obtained from the KCI mice as assessed by immunohistochemistry.

### NF-κB DNA binding activity was activated in KCI mice tissue

NF-κB has been reported to cross-talk with Notch pathway [28]. We have reported earlier that Notch-1 can up-regulate NF-κB DNA binding activity in pancreatic cancer [22]. Therefore, we investigated whether the downstream effect of Notch up-regulation could be mechanistically associated with the activation of NF-κB pathway in the tumors of these animals. It is well known that the NF-κB family is composed of homo- and heterodimers of Rel proteins; NF-κB1 (p50); NF-κB (p52), RelA (p65), RelB, and c-Rel (Rel). NF-κB (p50/p65) is a ubiquitous, constitutive and inducible heterodimer. In general, the DNA binding activity of NF-κB traditionally refers to the p50/p65 (p50/RelA) heterodimer-mediated binding to the DNA, and it is a known regulator of cell survival and anti-apoptosis signaling. In the nucleus, the p65 NF-κB subunit is a strong activator of a wide variety of genes; therefore, we assessed the nuclear expression of p65 protein by immunohistochemistry. Nuclear proteins from the tumors obtained from the transgenic mice were also subjected to NF-κB p65 ELISA, and NF-κB p65 DNA-binding activity as measured by EMSA. The results showed that the NF-κB p65 activity as assessed by ELISA, and the NF-κB p65 DNA binding activity was activated in tumors derived from the compound KCI mice (Fig. 2C, D). These results showed an increased nuclear accumulation of the p65 in the tumors of KCI mice, suggesting that both activation of K-ras and Ink4a/Arf deficiency are required for enhanced NF-κB activation. Moreover, immunostaining also showed that phospho-p65 was highly expressed in the nuclear compartment in the tumor tissues of KCI mice (Fig. 2D).

### NF-κB downstream genes are activated in KCI mice

It has been reported that Notch pathway stimulates NF-κB activity in cervical cancer cells by associating with the IKK signalosome through IKKα [29]. Previous study has shown that Notch pathway regulates the IKKα expression in pancreatic cancer [30]. Thus, we investigated the expression of IKK protein in the tumors of KCI mice. We found that all IKK family members such as IKKα, IKKβ and IKKγ were activated in the tumors of KCI mice (Fig. 3A). To further explore the effects of NF-κB activation, we examined the expression levels of certain NF-κB target genes including COX-2, cyclin D1, MMP-9, MMP-2, Bcl-2, c-myc, and survivin by real-time RT-PCR and western blotting, respectively, using the tumor tissues obtained from the compound KCI transgenic animals. Real-time RT-PCR and western blot analysis showed that the expression of these genes was activated in the tumors of KCI mice (Fig. 3A, B). We also found that the expression of Stat3 was activated in the tumors form KCI mice (data not shown). It is well known that these genes play critical roles in cell growth, invasion and metastasis. Therefore, these results further support the role of NF-κB in tumor growth and progression in the compound KCI mice.

**Figure 3:** The expression of Notch target genes is increased in KCI mice. **A,** Western blot analysis showing the up-regulated expression of IKK, p65, and NF-κB downstream genes in tumors derived from KCI mice. **B,** Real-time RT-PCR showing increased expression of NF-κB downstream genes such as survivin, cyclin D1, Bcl-2, C-myc, MMP-2, and MMP-9 in the tumors derived from the KCI mice. **C,** The expression of miR-200 family was down-regulated in the tumors of the KCI mice as assessed by real-time RT-PCR. **D,** Real-time RT-PCR showing decreased expression of E-cadherin, and increased expression of vimentin, and a modest increase in the expression of ZEB1 whereas a 30-fold increased expression of ZEB2 in tumors derived from the KCI mice.

### The miRNA-200 family was down-regulated in KCI mice

The miR-200 family have been found to regulate Notch signaling pathway [31]. The miR-200 family has five members: miR-200a, miR-200b, miR-200c, miR-141 and miR-429. We found that Notch-1 could be one of the target genes of miR-200 family (miR-200b, miR-200c) because over-expression of these miRNAs significantly inhibited Notch-1 expression in prostate cancer [31] and pancreatic cancer (unpublished data). To address whether miR-200 family is involved in the tumors of KCI mice which showed high expression of Notch (Notch-2 and 4) signaling pathway, we investigated the expression of miR-200 family. As expected, the expression of miR-200a, miR-200b and miR-200c was significantly decreased in the tumors of KCI mice (Fig. 3C). These results suggest that the tumors developed in the compound mice could show aggressive behavior such the acquisition of epithelial-to-mesenchymal transition (EMT) phenotype, and thus we have further investigated the molecular make-up of the tumors derived from the compound KCI transgenic mice as detailed below.

### Evidence of EMT phenotype in the tumors derived from the compound KCI transgenic mice

Recently many studies have shown that the miR-200 family regulates EMT by targeting zinc-finger E-box binding homeobox 1 (ZEB1) and ZEB2. EMT is a process by which epithelial cells undergo remarkable morphological changes characterized by a transition from epithelial cobblestone phenotype to elongated fibroblastic phenotype. Our previous studies have shown that miR-200a, miR-200b, and miR-200c were down-regulated in gemcitabine-resistant pancreatic cancer cells, consistent with the observed EMT phenotype [32], [33]. Furthermore, we have shown that miR-200 family regulates the expression of ZEB1, slug, E-cadherin, and vimentin, and thus suggested the re-expression of miR-200 could be useful for the reversal of EMT phenotype to mesenchymal-to-epithelial transition (MET), which has been partly documented in our recent publication [34]. Since we found low expression of miR-200 family in the tumors of KCI mice, we assessed the EMT markers to investigate whether the tumors in the KCI mice underwent EMT or not. We found loss of E-cadherin expression and elevated expression of vimentin and ZEB2 in the tumors of KCI mice although the expression of ZEB1 showed modest increase (Fig. 3D), suggesting that the expression of these factors may be important to induce EMT phenotype in the tumors of the KCI mice, which appears to be consistent with the aggressive behavior of the tumors developed in the compound KCI transgenic mice.

### Inhibition of Notch pathway caused reduced cancer cell growth in a mouse PDAC cell line

To further assess the potential role of Notch pathway in pancreatic cancer, we used Rink-1 cell line which was derived from the KCI pancreatic tissues and studied the effects of inhibitors of Notch pathway. Previous studies have shown that Rink-1 cells exhibited rapid growth *in vitro* and formed tumors in nude mice [14]. Since Notch signaling is activated *via* the activity of γ-secretase, several forms of γ -secretase inhibitors including DAPT and L-685,458 have been used to inactivate Notch pathway. Therefore, we determined the cell viability of Rink-1 cells treated with GSI by the MTT assay, and the data are presented in Figure 4A. The treatment of Rink-1 cells for 72 hours with DAPT, and L-685,458 resulted in cell growth inhibition. To determine which Notch receptor could be an effective therapeutic target for pancreatic cancer, the effect of Notch 1–4 siRNA on cell growth of the pancreatic cancer cells was examined. The efficacy of GSI and Notch siRNA for knockdown of Notch protein was confirmed through western blotting. We observed that Notch protein level was barely detectable in GSI treated or Notch siRNA transfected cells (Fig. 4B). Very interestingly, only inactivation of single Notch receptor did not significantly inhibit cell growth (Fig. 4A). These results suggest that inactivation of multiple Notch receptors by GSI are good way to treat PDAC. To confirm this conclusion, we tested the expression of Notch target genes in Rink-1 cells treated with GSI or Notch siRNA. Because only Notch-2 and Notch-4 siRNA slightly inhibited cell growth, we detected the expression of Notch target genes in Rink-1 cells treated with these two siRNAs. As we expected, we found that GSI inhibited the expression of Notch target genes including Hes-1, Survivin, Bcl-2, c-myc, uPA to more degree, compared to Notch-2 siRNA or Notch-4 siRNA transfection (Fig. 4C). Therefore, we used GSI in the following experiments. Next, we tested the effects of treatment on cell viability by clonogenic assay. GSI treatment resulted in a significant inhibition of colony formation of Rink-1 cells when compared with control (Fig. 5A). Overall, the results from clonogenic assay were consistent with the MTT data, suggesting that the inactivation of Notch pathway could inhibit cell growth of Rink-1 cells.

**Figure 4:** Inhibition of Notch pathway by Notch siRNA or GSI inhibited Rink-1 cell growth. **A,** Left panel, Inhibition of Rink-1 cell growth by Notch 1–4 siRNA tested by MTT assay. The results were plotted as means ± SD of three separate experiments having six determinations per experiment for each experimental condition. Middle and Right panel: L-685,458 and DAPT were γ-secretase inhibitors (GSI), which prevent the cleavage of the Notch receptor, blocking Notch signal transduction. GSI significantly inhibited Rink-1 cell growth. Cells were seeded in 96-well plates at 5,000 cells per well and treated with GSI for 72 hours. After treatment, cell densities were determined by MTT assay. Each value represents the mean ± SD (n = 6) of three independent experiments. *P<0.05, compared to the control. **B,** The expression of Notch pathway was down-regulated in Rink-1 cells treated with GSI or transfected with Notch 1–4 siRNA as assessed by western blotting analysis. **C,** The expression of Notch target genes was down-regulated in Rink-1 cells treated with GSI or transfected with Notch-2 siRNA or Notch-4 siRNA as assessed by as assessed by real-time RT-PCR.

**Figure 5:** GSI induced apoptosis, inhibited migration and invasion in Rink-1 cells. **A, Top,** Left panel: Cell survival of Rink-1 cells treated with GSI. Cells treated with GSI for 72 hours were evaluated by the clonogenic assay. Photomicrographic difference in colony formation in cells untreated and treated with GSI. Right panel: There was a significant reduction in the colony formation in Rink-1 cells treated with GSI compared with control cells. *P* values represent comparisons between cells treated with GSI and control using the paired *t* test. **Bottom,** Left panel: Characterization of apoptosis was carried out after propidium iodide (PI) and Annexin V-FITC staining with apoptosis detection kit followed by flow cytometric analysis after 48 h of GSI treatment of Rink-1 cells. The percentage of apoptotic cells increased from 10% in the control to 28–33% in GSI treated cells. Right panel: GSI induced apoptosis in Rink-1 cells. Rink-1 cells were exposed to GSI for 72 hours. Apoptosis was measured by Histone DNA ELISA. Values are reported as mean ± SD. *P<0.05, compared to the control. **B, Top,** Left panel, Invasion assay using GSI treated cells showing low penetration of cells through the Matrigel-coated membrane, compared with control cells. Right panel: The graphs showing the value of fluorescence from the invaded Rink-1 cells. The values indicate the comparative amount of invaded Rink-1 cells. **Bottom,** Wound healing assay was conducted to assess the capacity of cell migration. GSI treatment decreased the cell migration in Rink-1 cells. **C,** GSI inhibited the NF-κB DNA binding activity in Rink-1 cells as assessed by EMSA. **D,** Real-time RT-PCR and western blot analysis showed that L-685,458 inhibited the expression of Survivin, c-myc, Bcl-2, and uPA genes.

### Inhibition of Notch pathway caused apoptotic cell death in Rink-1 cell line

Next, we investigated whether the overall growth inhibitory effects of GSI are in part due to induction of apoptosis, which was examined by using an ELISA-based assay. These results provided convincing data that GSI induced apoptosis in Rink-1 cell line (Fig. 5A). To confirm these results, we also used annexin V-FITC method to detect the apoptosis induced by GSI for which Rink-1 cells were treated with GSI for 48 hours. By staining cells with annexin V-FITC and PI, FACS analysis was used to distinguish and quantitatively determine the percentage of dead, viable and apoptotic cells after treatment. We found that the percentage of apoptotic cells increased from 10% in the control to 28–33% in Rink-1 cells after GSI treatment (Fig. 5A). These results provided convincing data showing that inactivation of Notch pathway could induce apoptosis in Rink-1 pancreatic cancer cells.

### Inhibition of Notch pathway decreased cancer cell migration and invasion

Notch pathway is believed to be critically involved with the processes of tumor cell invasion and metastasis. Previous studies have shown that pancreatic tumors arising in the compound KCI mice have extensive invasion of adjacent organs, including the duodenum, stomach, liver, and spleen [13]. In order to better understand whether Notch pathway has a critical role in invasion, we tested the effects of inactivation of Notch pathway on cancer cell invasion. We found that GSI treated cells showed a lower level of penetration through the matrigel-coated membrane compared with the control cells. The value of fluorescence from the invaded Rink-1 cancer cells was decreased about 5–7 fold compared with that of control cells (Fig. 5B). In order to further examine the effect of GSI on cell migration and invasion, we conducted wound healing assay in Rink-1 cells. The results show that GSI treatment inhibited the capacity of wound healing in Rink-1 cells (Fig. 5B), suggesting that GSI can inhibit cell migration and invasion. These results suggest a direct role of Notch signaling in Rink-1 cancer cell migration and invasion, and these results are consistent with aggressiveness of tumors developed in the compound KCI transgenic animal.

### Inhibition of Notch pathway decreased NF-κB DNA-binding activity

We investigated whether the downstream effect of Notch-1 down-regulation was mechanistically associated with the NF-κB pathway. Nuclear proteins from GSI treated cells were subjected to analysis for NF-κB p65 DNA-binding activity as measured by EMSA. The results showed that GSI significantly inhibited NF-κB p65 DNA-binding activity compared to control (Fig. 5C). These results provided evidence in support of a mechanistic crosstalk between Notch and NF-κB in pancreatic cancer. Furthermore, we also found that GSI inhibited NF-κB downstream gene expression, such as Survivin, Bcl-2, c-myc, and uPA (Fig. 5D).

### Over-expression of miR-200b inhibited the cell growth through Jagged ligands

Recently, it has been reported that miR-200 family members target Notch pathway components, such as Jagged-1 [35], [36]. In order to examine whether miR-200 family regulate Notch pathway, we transfected miR-200b precursor into Rink-1 cells. We confirmed that the transfection of miR-200b precursor increased the relative level of miR-200b in Rink-1 cells (Fig. 6A). Over-expression of miR-200b decreased the relative mRNA levels of Jagged-1, Jagged-2 and their target genes by real time RT-PCR assay (Fig. 6A). The data from western blot analysis demonstrated that over-expression of miR-200b decreased the relative protein levels of Jagged-1 and its target gene such as Hes-1, Hey-1, and Bcl-2 (Fig. 6B). Moreover, we found that over-expression of miR-200b inhibited cell growth in Rink-1 cells (Fig. 6B). Next, we detected whether inhibition of Jagged-1 could inhibit cell growth. Jagged-1 siRNA significantly decreased the expression of Jagged-1 and its target Hes-1 and Hey-1 at mRNA and protein levels (Fig. 6C). Furthermore, we found that inhibition of Jagged-1 by Jagged-1 siRNA inhibited the Rink-1 cell growth (Fig. 6C), suggesting that Jagged-1 could be a potential target for pancreatic cancer.

**Figure 6:** The miR-200b inhibited Rink-1 cell growth and Jagged-1 expression. **A,** Left panel, Re-expression of miR-200b was established in Rink-1 cells by transfection with its precursor. Middle panel, Re-expression of miR-200b did not regulate the expression of Notch receptors in Rink-1 cells. Right panel, Re-expression of miR-200b regulated the expression of Jagged-1 and Jagged-2 mRNAs in Rink-1 cells. **B,** Left and middle panel, Re-expression of miR-200b inhibited the expression of Jagged-1 target genes at mRNA and protein levels in Rink-1 cells. Right panel, Re-expression of miR-200b inhibited Rink-1 cell growth test by MTT assay. **C,** Left and middle panel, Jagged-1 siRNA inhibited the expression of Jagged-1 target gene Hes-1 and Hey-1 at mRNA and protein levels in Rink-1 cells. Right panel, Jagged-1 siRNA inhibited Rink-1 cell growth test by MTT assay.

## Discussion

PDAC is the fourth leading cause of cancer-related deaths in the United States [1]. Although some progress in chemotherapy, radiation therapy, and surgical technique, the overall survival rate for five years is less 4% of all patients diagnosed with PDAC [1]. These disappointing outcomes suggest that new and alternative approaches to the understanding the mechanisms of PDAC progression is critically needed. Transgenic mice are good models to identify the pathogenic role of specific gene mutations and core signaling pathways associated with pancreatic cancer.

It has been known that K-ras mutations are observed in 80%–90% of pancreatic cancer. Oncogenic K-ras is involved in the initiation or early stages in the development of PDAC. Therefore, the conditional KC mice are considered good tools for mechanistic studies of pancreatic cancer progression. Since KC mice mimic slow progression from PanIN to invasive cancer in around 12–15 months [6], [37], but the KC mice bred with many other transgenic mice showed rapid development the PDAC. For example, Smad4/Dpc4 haploinsufficiency shortened the life span of KC mice to median survival of approximately 8 months [10]. LSL- K-ras^G12D^; Pdx1-Cre; Trp53R mice have a dramatically shortened median survival of approximately 5 months [6]. The median survival time of KC mice with LKB1 heterozygosity was 4.5 months [11]. PTEN haploinsufficiency significantly shortened the life span of KC mice to a median survival of around 3.5 months [9]. The p21 heterozygosity made the KC mice with a median survival of 2.5 months [11]. One mouse model having activated K-ras and Ink4a/Arf deficiency had median survival of 2 months [13]. Therefore, for the present study, we used the compound KCI mice (activated K-ras and Ink4a/Arf deficiency) to investigate the mechanisms of pancreatic cancer progression.

Pancreatic cancer has been shown to have deregulated Notch signaling pathway. Although Notch pathway has been reported to have a tumor suppressive role in certain specific condition [18], the majority of studies show that the activated Notch pathway contributes to PDAC tumorigenesis [19], [25], [38]–[40]. The high level expression of Notch receptors, Notch ligands and Notch target genes have also been observed in human pancreatic cancer [19]–[21], [38]–[40]. Notch activity is required for TGF-α-induced acinar-to-ductal transition and prevention of Notch activation by GSI prevents acinor-to-ductal metaplasia in TGF-α-treated cells [41]. It has been reported that GSI inhibited tumor progression in LSL-K-ras^G12D^; Pdx1-Cre; Trp53R mouse model of PDAC [24]. Moreover, it has been found that Notch signaling was downstream of K-ras gene in pancreatic cancer [23], [42]–[44]. In this study, we used the compound KCI mice, which recapitulated most features of human pancreatic cancer to determine whether Notch signaling could be required for the development of PDAC. Indeed, we found over-expression of Notch signaling pathway in the tumors of KCI mice. The molecular explanation for the high expression of Notch in the tumors of KCI mice could be due to Ink4a/Arf deficiency. Furthermore, inhibition of Notch pathway by GSI in murine pancreatic cancer cell line Rink-1 inhibited cell growth, migration, and invasion, suggesting that Notch signaling pathway appears to be a viable therapeutic target for PDAC, which has been an active area of drug development.

The cross-talk between Notch and NF-κB in PDAC has been found in human cancer including pancreatic cancer [22], [28], [45]. It was found that Notch pathway stimulated NF-κB activity in cervical cancer cells by associating with the IKK signalosome through IKKα [29], [46]. We have reported that Notch pathway can regulate NF-κB activity in pancreatic cancer [21], [22]. In the present study, we found that NF-κB was activated in the tumors of KCI mice, suggesting that the downstream effect of Notch pathway up-regulation was mechanistically associated with the activation of NF-κB signaling pathway in the tumors developed in the compound KCI transgenic mice. Moreover, activated NF-κB-regulated genes which are involved in cell growth, apoptosis, migration, and invasion are also activated. Furthermore, GSI inhibited NF-κB activity and its downstream genes in Rink-1 cells. These results demonstrate the importance of NF-κB signaling and provide a basis to consider the pharmacological inhibition of the NF-κB for the treatment of PDAC, which has also been an active area of drug development.

In recent years, microRNAs (miRNAs) have been reported to participate in Notch pathway regulation in pancreatic cancer [47]. One important miRNA is miR-200 family, which is involved in the regulation of EMT, stem cells and the regulation of Notch pathway [35], [36]. The miR-200 family has five members: miR-200a, miR-200b, miR-200c, miR-141 and miR-429. Our previous study has shown that Notch pathway could be one of the target of miR-200b [31]. Consistent with this notion, we found loss of miR-200a, miR-200b, and miR-200c expression in the tumors of KCI mice, suggesting that activated Notch pathway could also be due to the loss of expression of miR-200 family. Over-expression of miR-200b decreased the expression of Jagged ligands and Notch target gene such as Hes-1, Hey-1, and Bcl-2, leading to cell growth inhibition. Moreover, we found that over-expression of miR-200b inhibited cell growth in Rink-1 cells (Fig. 6B). Most interestingly, recent studies have shown that the miR-200 family regulates EMT by targeting ZEB expression. We have reported earlier that miR-200a, miR-200b, and miR-200c are down-regulated in gemcitabine-resistant pancreatic cancer cells, which have high expression of Notch pathway and contributed to the acquisition of EMT phenotype [33], [34]. The acquisition of EMT has been documented to be involved with invasion and metastasis, and thus our data on the loss of miR-200 suggest that the EMT phenotypic tumors in our compound mice, and that the tumors in these animals are invasive and metastatic compared to pancreata with K-ras activation or Ink4a/Arf loss alone.

Based on our results, we conclude that one possible mechanism by which the tumors developed in the compound KCI transgenic mice with activated K-ras and Ink4a/Arf deficiency is in part due to the loss of miR-200 family, which leads to the activation of Jagged/Notch and NF-κB signaling pathway, resulting in the up-regulation of NF-κB target genes, such as MMP-9, c-myc, survivin, Bcl-2, cyclin D1, and COX-2 as summarized in the cartoon diagram (Fig. 7) and contributes to tumor aggressiveness. Although we have demonstrated the loss of miR-200, and the activation of Notch and NF-κB signaling pathway in the current animal model; however, there maybe other genetic alterations causing tumor aggressiveness in this compound mice with activated K-ras and Ink4a/Arf deficiency, suggesting that further in-depth studies are needed to investigate the precise molecular mechanism of tumor progression in this mouse model. Moreover, novel strategies for the re-expression of miR-200 and its consequence could be tested in this animal model, which would help in the rational drug design in addition to Notch and NF-κB targeted drugs for the treatment of human PDAC for improving the overall survival of patients diagnosed with this devastating disease.

**Figure 7:** The schematic representation of our proposed molecular mechanism involved in the development and progression of tumors in the compound KCI transgenic mice.

## Materials and Methods

### Ethics Statement

This study was carried out in strict accordance with the recommendations in the Guide for the Care and Use of Laboratory Animals of the National Institutes of Health. Any animal found unhealthy or sick were promptly euthanized. The protocol was approved by the Committee on the Ethics of Animal Experiments of Wayne State University institutional Users Animal Care Committee (Permit Number: A-10-03-08).

### Mouse Model

The LSL-K-ras^G12D^ strain was bred to the following strains: Pdx1-Cre, INK4a/Arf ^lox/lox^ as previously described [14], [48]. Pancreata were collected and processed for further analysis.

### Genotyping

For genotyping, genomic DNA was extracted from tail cuttings using the REDExtract-N-Amp Tissue PCR kit (Sigma-Aldrich, St. Louis, Missouri). Three PCR reactions were carried out for each animal to investigate the presence of the oncogenic K-ras, p16 and Pdx1-Cre transgenes, respectively.

### Cell lines

Rink-1 murine pancreatic tumor cell line was generated from the pancreatic tissue obtained from LSL- Kras^G12D^; Pdx1-Cre; Ink4a/Arf mice as previously described [13], [14].

### Histopathology and immunohistochemistry

Histopathologic analysis of pancreata was carried out. The expression of Ki-67, Notch, and phospho-p65 was assessed in histological sections of tumors as described before [49].

### Real-time reverse transcription-PCR analysis for gene expression studies

The total RNA from animal tissues was isolated by Trizol (Invitrogen, Carlsbad, CA) according to the manufacturer's protocols. The primers used in the PCR reaction were described earlier [21], [22], [31], [50]. Real-time PCR amplifications were performed as described earlier [21].

### Western blot analysis

The animal tissues were homogenized and sonicated in 62 mM Tris-HCl and 2% SDS. In another set of experiments, cytoplasmic and nuclear proteins were also extracted. The proteins were used for western blotting as described earlier [21].

### Electrophoretic mobility shift assay (EMSA)

Nuclear extracts were prepared from animal tissues and electrophoretic mobility shift assay was done by incubating 10 µg nuclear extract with IRDye-700-labeled NF-κB oligonucleotide as described earlier [22].

### NF-κB p65 DNA-binding activity assay

Nuclear extracts (5 µg) was used to determine p65 DNA-binding activity using an enzyme-linked immunosorbent assay (ELISA)-based assay according to the manufacture's instructions (Active Motif TransAM).

### TaqMan miRNA real-time reverse transcription–PCR

To determine the expression of miRNAs in transgenic mice tissues, we used TaqMan miRNA assay kit (Applied Biosystems) following manufacturer's protocol. Total RNA was extracted, and 5 ng from each sample were reverse transcribed as described earlier [32]. Real-time PCR reactions were then carried out in a total volume of 25 µL reaction mixture using Smart Cycler II (Cepheid) as described earlier [32].

### Cell invasion assay

The invasive activity of the cells was tested using the BD BioCoat Tumor Invasion Assay System (BD Biosciences, Bedford, MA) as described earlier [22].

### Wound healing assay

Wound healing assay was conducted to examine the capacity of cell migration. Briefly, the wound was generated in the cells with 90–95% confluent by scratching the surface of the plates with a pipette tip. The cells were then incubated in the absence and presence of GSI for 24 h, and then photographed with a Nikon microscope.

### siRNA, miRNA and transfection experiments

Cells were transfected with 100 nmol/L of Notch-1, Notch-2, Notch-3, Notch-4, Jagged-1 siRNA or control siRNA (Santa Cruz) as well as 20 nmol/L of miR-200b (Ambion, Austin, TX) using DharmaFECT3 siRNA transfection reagent (DHARMACON, Lafayette, CO) as previously described [31].

### Densitometric and statistical analysis

The statistical significance of differential findings between experimental groups and control groups was statistically evaluated using GraphPad StatMate software (GraphPad Software, Inc., San Diego, CA). *P* values lower than 0.05 were considered statistically significant.
